This article has been retracted.

# Quercetin Prevents Radiation-Induced Oral Mucositis by Upregulating BMI-1

**DOI:** 10.1155/2021/2231680

**Published:** 2021-11-27

**Authors:** Jing Zhang, Yiyang Hong, Zhenyu Liuyang, Haozhe Li, Zhongyang Jiang, Jingjing Tao, Hai Liu, Anyong Xie, Yili Feng, Xingjian Dong, Yihong Wang, Qinghua Dong, Guanyu Wang

**Affiliations:** ^1^Biomedical Research Center, Sir Run Run Shaw Hospital, School of Medicine, Zhejiang University, Hangzhou, 310016 Zhejiang, China; ^2^Department of General Surgery, Sir Run Run Shaw Hospital, School of Medicine, Zhejiang University, Hangzhou, 310016 Zhejiang, China; ^3^Department of Radiotherapy, Sir Run Run Shaw Hospital, School of Medicine, Zhejiang University, Zhejiang, 310016 Hangzhou, China; ^4^Institute for Translational Medicine, School of Medicine, Zhejiang University, Zhejiang, 310016 Hangzhou, China; ^5^College of Life Science and Technology, Huazhong Agricultural University, Wuhan, 430070 Hubei, China; ^6^Department of Pathology, Sir Run Run Shaw Hospital, School of Medicine, Zhejiang University, Hangzhou, 310016 Zhejiang, China; ^7^Key Laboratory of Cancer Prevention and Intervention, China National Ministry of Education, Hangzhou, 310009 Zhejiang, China

## Abstract

Radiation-induced oral mucositis is a major adverse event of radiotherapy. Severe oral mucositis may cause unwanted interruption in radiotherapy and reduce long-term survival in cancer patients receiving radiotherapy, but until now, there have been no effective options for preventing radiation-induced oral mucositis. Quercetin is a flavonoid that is widely found in food species and has anti-inflammatory, antioxidant, and anticancer activities. In this study, we investigated a new role of quercetin in preventing radiation-induced oral mucositis. Quercetin exerted preventive effects against radiation-induced oral mucositis induced by single-dose (25 Gy) ionizing radiation or fractionated ionizing radiation (8 Gy × 3) in C57BL/6 mice and maintained the proliferation ability of basal epithelial cells. Quercetin pretreatment alleviated reactive oxygen species generation, NF-*κ*B pathway activation, and downstream proinflammatory cytokine production and reduced DNA double-strand breaks and cellular senescence induced by ionizing radiation. Quercetin also upregulated BMI-1 expression in oral epithelial cells and promoted ulcer repair. In addition, quercetin exerted similar radioprotective effects in irradiated primary cultured normal human keratinocytes, reduced reactive oxygen species generation and proinflammatory cytokine release, and promoted DNA double-strand break repair and wound healing by upregulating the expression of BMI-1, which is a polycomb group protein. Thus, quercetin can block multiple pathological processes of radiation-induced oral mucositis by targeting BMI-1 and may be a potential treatment option for preventing radiation-induced oral mucositis.

## 1. Introduction

Radiation-induced oral mucositis (RIOM) is a major dose-limiting acute side effect of radiotherapy (RT) in cancer patients. In particular, almost all head and neck cancer (HNC) patients receiving RT develop RIOM [1]. RIOM is painful and induces weight loss, odynophagia, and secondary infections. Severe RIOM can lead to hospitalization and the requirement for a feeding tube, which may cause unwanted interruption in RT and reduce long-term survival [2].

A five-phase model has been accepted to explain the pathogenesis of RIOM, involving initiation, primary damage, signaling amplification, ulceration, and healing phases [3]. The initiation phase results in DNA strand breaks and reactive oxygen species (ROS) generation. In the primary damage phase, nuclear factor-*κ*B (NF-*κ*B) is activated and proinflammatory cytokines (IL-6, IL-1*β*, TGF-*β*, TNF-*α*, etc.) are released. During the phase of signaling amplification, increased inflammatory factors exaggerate the expression of genes regulated by NF-*κ*B and already existing inflammation. This leads to ulceration and epithelial loss, and the basement membrane is disrupted. In the healing stage, the oral mucosal epithelium reepithelializes to promote ulcer healing. Until now, there have been no effective options for preventing RIOM in cancer patients receiving RT [4]. The main preventive method for RIOM in the clinic is maintaining good oral care. Palifermin, a truncated human keratinocyte growth factor, is the only FDA-approved drug for preventing oral mucositis in leukemia patients who receive bone marrow transplantation [5]. Clinical trials have shown that palifermin has a modest preventive effect against severe oral mucositis in HNC patients undergoing postoperative radiochemotherapy [6]. Thus, the identification of new agents that can prevent RIOM is critical to improve the quality of life of cancer patients receiving RT.

Quercetin (3,3′,4′,5,7-pentahydroxyflavone) is a flavonoid widely found in food. Quercetin has anti-inflammatory, antioxidant, antibacterial, and anticancer activities [7, 8]. Although the mechanisms are largely unknown, studies have shown that quercetin can attenuate radiation-induced bladder, lung, neuron, and kidney damage [9–11], inhibit radiation-induced colon colitis [12], and mitigate radiation-induced skin fibrosis [13]. Therefore, we hypothesize that quercetin may play a radioprotective role in the oral mucosa. In this study, we investigated the preventive effects of quercetin in irradiated mice and primary cultured normal human keratinocytes (NHKs).

## 2. Methods and Materials

### 2.1. Experimental RIOM Mouse Model

Twenty-five adult (6–8 weeks old) female C57BL/6 mice (Slaccas, Shanghai) were randomly divided into five groups (*n* = 5): no IR, S-IR (p.o. PBS, 25 Gy IR), F-IR (p.o. PBS, 8 Gy × 3 IR), S − IR + QCT (p.o. quercetin, 25 Gy IR), and F − IR + QCT (p.o. quercetin, 8 Gy × 3 IR).

#### 2.1.1. Animal Irradiation

After weighing, we anesthetized the mice with ketamine (80 mg/kg, i.p.) and xylazine (12 mg/kg). The head and neck of the mouse were exposed to IR delivered with a precision X-ray irradiator (X-RAD 160, PXi, USA), and the rest of the body was covered with a lead plate. Mouse RIOM was induced by a single dose (S-IR, 25 Gy) or fractionated cranial irradiation (F-IR, 8 Gy/day for 3 days, accumulative to 24 Gy). No IR mice were anesthetized but not exposed to radiation.

#### 2.1.2. Quercetin Treatment

Quercetin was obtained from Sigma (MO, USA). Mice were pretreated with quercetin (p.o. 300 mg/kg, once daily) for 7 days before IR, and the treatment continued for 8 days after IR.

The day of IR was designated as day 1. We monitored irradiated mice and checked their body weights daily. Mice were sacrificed on day 9. Mouse tongues were harvested and stained with 1% toluidine blue (TB). Increased TB staining indicated the severity of oral mucositis. Then, tongues were collected for immunochemistry (IHC), hematoxylin & eosin (HE) staining, and further analysis of protein and RNA expression.

### 2.2. NHK Culture and Treatment

The isolation of primary NHKs from foreskin and the culture of NHKs were described previously [14]. To obtain NHK/control and NHK/shBMI-1 cells, we infected NHKs (passage 1) with lentivirus carrying a control vector (GCSIL-GFP) or BMI-1 shRNA (GCSIL-GFP-sh*BMI-1*) purchased from GeneChem (Shanghai). NHKs (passage 2 or 3) were pretreated with 20 *μ*M quercetin for 2 h before IR using an X-RAD 160 irradiator.

### 2.3. Western Blot Analysis

Immunoblotting was performed as described in our previous study [14]. Briefly, mouse tongues and NHKs were treated with RIPA buffer. The supernatant was subjected to SDS–PAGE and transferred to PVDF membranes. The membrane was incubated with the antibodies listed in Table S1 and photographed in ChemiDoc (Bio-Rad, USA).

### 2.4. Quantitative Real-Time PCR (qPCR)

Total RNA was extracted using TRIzol Reagent (Invitrogen, CA), and reverse transcription was performed using cDNA Synthesis SuperMix (Vazyme, China) according to the manufacturer's instructions. qPCR of each sample was performed three times using 2 × SYBR Green QPCR Master Mix (Biomarker, USA) and was detected in the ViiA 7 Real-Time PCR System (Life Technologies, NY, USA). Primers were obtained from Sangon (Shanghai, China). The primer sequences are listed in Table S2.

### 2.5. Immunohistochemistry and Immunofluorescence

The paraffin sections were stained using standard immunohistochemical procedures. Sections were incubated with anti-Ki67, anti-BMI-1, anti-*γ*-H2AX, anti-8-OHDG, and anti-p-p65 antibodies as indicated in Table S1. We performed immunofluorescence staining (IF) using anti-p-*γ*-H2AX as the primary antibody and a secondary antibody conjugated to Cy3 (Jackson ImmunoResearch, USA). The nuclei were stained with DAPI (Solarbio, China).

### 2.6. Colony Formation Assay

NHKs were plated in 6-well plates at 500–30000 cells per well, pretreated with 20 *μ*m quercetin for 2 h, and then irradiated with 0, 2, 4, 6, 8, or 10 Gy. After irradiation, the cells were cultured for another 10 days and then stained with 0.5% crystal violet and the colonies were counted to calculate the sensitization enhancement ratio (SER).

### 2.7. Cellular Senescence Activity Assay

NHKs were washed with PBS and fixed at room temperature in 2% formaldehyde and 0.2% glutaraldehyde solution for 15 min. Then, NHKs were stained with senescence-associated *β* galactosidase (SA-*β*-Gal) staining solution (Beyond Biotech, China) and incubated overnight at 37°C according to the instructions of Beyond Biotech (Hangzhou, China).

### 2.8. Tissue and Intracellular ROS Assays

Fresh frozen sections were incubated with 5 *μ*M dihydroethidium (DHE) (Beyotime Biotech, China), and then, the nuclei were stained with DAPI. The samples were imaged with an AXIO Observer A1 inverted fluorescence microscope (Carl Zeiss, Germany). NHKs were stained with DHE, and then, the fluorescence intensity of DHE was detected using a FACSCalibur (Becton Dickinson, San Jose, CA) and analyzed in CellQuest software.

### 2.9. Neutral Comet Assay

We performed a neutral comet assay to detect DNA double-strand breaks (DSBs) using a comet assay kit (Trevigen, Gaithersburg, MD, USA) according to the manufacturer's instructions. After pretreatment with 20 *μ*m quercetin for 2 h, NHKs were exposed to 5 Gy IR, harvested at 6 h post-IR and then placed on comet slides. Neutral comet electrophoresis was performed and then stained with Gel Red (Biotium, USA). Images were obtained with a laser confocal microscope (TCS SP8, Leica, Germany). The tail length was measured by the Comet Analysis Software Project (CASP) to compare the DSBs in NHKs.

### 2.10. Homology-Directed Repair of DNA and Quantification of Nonhomologous End Joining (NHEJ) Events

As previously described [15], 10 *μ*g of AAVS1-sgRNA plasmid, 10 *μ*g of pMD2G plasmid, and 10 *μ*g of pspax2 plasmid were transfected into 239T cells with LipoFilter (HanBio, Shanghai, China). To analyze the insertion/deletion patterns in NHEJ products, NHKs were infected with AAVS1-sgRNA lentivirus produced by 239T cells. After purification by puromycin, NHKs were pretreated with DMSO or 50 *μ*M quercetin for 2 h, the medium was changed to 20 *μ*M quercetin, and the cells were infected with U6-Cas9-EGFP lentivirus purchased from GeneChem (Shanghai, China). NHKs were collected after CRISPR/Cas9-induced NHEJ. gDNA was isolated from NHKs using a genomic DNA purification kit (TIANGEN). The genomic regions of 300–500 bp surrounding the CRISPR/Cas9 target sites were PCR amplified with AAVS1 primers. PCR products were purified using a gel extraction kit (TIANGEN). As NHEJ in normal cells generates deletions mostly within ∼50 bp, PCR products of 300–500 bp are expected to cover most NHEJ products. For next-generation sequencing at Novogene Co. Ltd. (Beijing), the PCR products were cleaned, quantified, normalized into one library pool, and sequenced on an Illumina HiSeq. After demultiplexing, forward and reverse paired-end reads were merged to generate a single consensus sequence per read pair using PEAR 0.9.8. Merged sequences were analyzed using the “DeepSeq Pipeline,” a self-analysis platform programmed by Xie's lab. “Deletion” sequences were determined by gaps (dashes) in the read sequence.

### 2.11. Wound Healing

NHKs were inoculated in a 6-well plate (5 × 10^5^ cells/well) until the monolayer reached a degree of fusion of 80–90%, after which it was scratched with the tip of a pipette. NHKs were exposed to 5 Gy IR after quercetin pretreatment for 2 h. Photos were taken at 24 h and 48 h post-IR.

### 2.12. Statistical Analysis

Differences among groups were analyzed by Student's two-tailed *t*-test or one-way ANOVA. Differences with *P* < 0.05 were considered significant. Data were expressed as the mean ± SEM. A two-tailed Mann–Whitney test was used to analyze NHEJ between the two groups.

## 3. Results

### 3.1. Quercetin Prevents Radiation-Induced Ulcer Formation

To test the protective effect of quercetin on the oral mucosa, we generated S-IR- and F-IR-induced RIOM mouse models that mimic clinical RIOM development. The overall situation of the mice was observed, and the daily changes in body weight were recorded after IR. As a result of inadequate food and water intake, the irradiated mice showed significant reductions in activity, weakness, and body weight of approximately 36% and 42% in the S-IR and F-IR groups, respectively. In contrast, mice pretreated with quercetin showed less weight loss after IR (Figure 1(a)). S-IR and F-IR caused RIOM ulcer formation mainly on the back of the tongue base, the ulcer was stained deep blue, and the average size of the ulcer was 1.96 mm in both S-IR and F-IR mice. Quercetin significantly attenuated the formation of ulcers and reduced the size of ulcers to 0.18 mm at day 9 after IR (Figures 1(b) and 1(c)). HE revealed that the integrity of the mucosa was lost, the layered squamous epithelium had completely disappeared, and many inflammatory cells had infiltrated the irradiated tissues. In mice pretreated with quercetin, due to the influence of irradiation, the epithelial stratification structure was slightly disordered and the epithelium became thinner compared with that of no IR mice, but the integrity of the mucosa was still maintained (Figure 1(d)). These results suggest that quercetin has a preventive effect against S-IR- and F-IR-induced tongue mucosal injury.

### 3.2. Quercetin Maintains Cell Proliferation and Reduces Cellular Senescence after IR

Previous studies have shown that IR can induce depletion of epithelial stem cells, which are essential for mucosal proliferation and renewal [16]. Ki-67 is a classic marker of cell proliferation; therefore, we detected the expression of Ki-67 in the basal layer of the oral mucosa. Ki-67 expression was abundant in the basal layer of the oral mucosa not exposed to radiation. Due to IR damage to the epithelium, the number of Ki-67-positive cells had sharply decreased in the irradiated oral mucosa. Quercetin-pretreated mice showed no obvious decrease in the number of Ki-67-positive cells compared with no IR mice (Figure 2(a)). PCNA is another good indicator of the cell proliferation status. Consistent with the IHC results, S-IR and F-IR decreased PCNA protein expression in irradiated mouse tongues. The PCNA expression level in quercetin-pretreated mice was similar to that in no IR mice (Figure 2(b)). IR-induced premature senescence in basal epithelial cells is associated with the pathogenesis of RIOM. The protein expression of IR-induced p21, a well-known marker of cellular senescence, was inhibited in quercetin-pretreated mouse tongues (Figure 2(c)). The mRNA expression levels of p21 and p16^INK4A^, another marker of senescence, were markedly increased after IR. Quercetin pretreatment notably inhibited the transcript expression of both p16^INK4A^ and p21 in S-IR and F-IR mouse tongues (Figure 2(d)).

The basal epithelial cells in the oral mucosa are mainly keratinocytes. We further investigated the effects of quercetin *in vitro* using primary human NHKs. Quercetin had no toxic effect on NHKs and promoted NHK proliferation after 24 h of treatment at 2.5–20 *μ*M (Figure S1); therefore, we selected a 2 h pretreatment with 20 *μ*M quercetin. Irradiated senescent NHKs became enlarged with a flattened morphology and showed irreversible loss of proliferative activity. Quercetin pretreatment reduced the number of SA-*β*-gal-positive NHKs at days 3, 5, and 7 after IR, which means that less cellular senescence occurred (Figures 2(e) and 2(f)). To evaluate the radiation response of NHKs affected by quercetin, we performed a colony formation assay. Significantly, more colonies formed in the quercetin-pretreated NHKs than in the irradiated control NHKs (Figure 2(g)), indicating that quercetin pretreatment increased cell proliferation and reduced the radiosensitivity of NHKs, with an SER of 0.58 (Table S3). Similar to the *in vivo* results, quercetin pretreatment maintained PCNA expression and inhibited IR-induced p21 expression in NHKs after IR (Figure 2(h)). These *in vivo* and *in vitro* results demonstrate that quercetin pretreatment can effectively reduce IR-induced cellular senescence and maintain cell proliferation.

### 3.3. Quercetin Attenuates IR-Induced ROS Generation

In the initial phase of RIOM, RT rapidly causes direct and lethal DNA damage with the release of ROS from epithelial cells. Therefore, we first investigated the effects of quercetin on ROS generation *in vivo*. S-IR and F-IR induced significant increases in DHE fluorescence not only in oral epithelial cells but also in fibroblasts under the epithelium, demonstrating that IR induced a large amount of intracellular ROS production (Figure 3(a)). Quercetin pretreatment dramatically inhibited ROS production, as indicated by the reduced oral fluorescence. 8-OHDG is produced by deoxyguanosine in DNA by ROS and can be used to evaluate the degrees of oxidative damage and repair *in vivo* [17]. In irradiated oral mucosa, a significant increase in 8-OHDG expression was observed at day 9 after IR but quercetin pretreatment reduced its expression (Figure 3(b)). p47 is an important NADPH oxidase in ROS production and was significantly induced by S-IR and F-IR. Accordingly, quercetin pretreatment obviously inhibited the increase in p47 expression in irradiated mouse tongues (Figure 3(c)). We then investigated the effect of quercetin on ROS generation in NHKs after IR. Quercetin pretreatment also effectively attenuated IR-induced total ROS generation (Figures 3(d) and 3(e)) and reduced p47 expression in NHKs after IR (Figure 3(f)).

### 3.4. Quercetin Promotes DNA Repair after IR

To examine the potential role of DNA repair in the preventive effects of quercetin against RIOM, we detected DNA double-stranded break (DSB) formation by staining for *γ*-H2AX. The number of *γ*-H2AX-positive cells was markedly increased in S-IR and F-IR mouse tongues but significantly lower in quercetin-pretreated mouse tongues, indicating that quercetin pretreatment attenuated IR-induced DNA DSB formation (Figure 4(a)). Consistent with the *γ*-H2AX IHC results, the protein levels of *γ*-H2AX in quercetin-pretreated mouse tongues were significantly reduced compared with those in S-IR and F-IR mouse tongues (Figure 4(b)).

We then investigated whether quercetin affects DSB repair in NHKs after IR. NHKs were stained to identify *γ*-H2AX foci, an indicator of DSB number. The number of *γ*-H2AX foci was markedly increased in irradiated NHKs but was greatly reduced in quercetin-pretreated NHKs (Figure 4(c)). Meanwhile, the protein levels of *γ*-H2AX in quercetin-pretreated NHKs were reduced at days 2 and 5 after IR compared with irradiated NHKs (Figure 4(d)). Comet assays showed that irradiated NHKs had much longer comet tails than nonirradiated NHKs, but quercetin-pretreated NHKs showed much shorter comet tails after IR, indicating fewer DSBs in quercetin-pretreated NHKs than in irradiated NHKs (Figure 4(e)). Furthermore, we analyzed the deletion length of the nonhomologous end joining (NHEJ) products to gain a better understanding of the role of quercetin in promoting DNA-directed repair. Compared with the control NHKs, deletions in quercetin-pretreated NHKs were shifted toward shorter lengths. The median deletion lengths were 1 bp in quercetin-pretreated NHKs and 4 bp in control NHKs (Figure 4(f)), and over 85% of the deletion length of quercetin-pretreated NHKs was less than 1 bp (Figure 4(g)). These results suggest that quercetin mitigates IR-induced DNA damage and promotes DNA repair.

### 3.5. Quercetin Inhibits NF-*κ*B Activation and Proinflammatory Cytokine Production Induced by IR

During the signaling and amplification phases of RIOM, ROS and DNA damage trigger the activation of the NF-*κ*B pathway and promote the production of a large number of proinflammatory factors, which restimulate NF-*κ*B activation and then produce more cytokines. To investigate whether quercetin affects NF-*κ*B activation, we checked phosphorylated NF-*κ*B (p-p65) expression in mouse tongues. The basal layer cells of oral mucosa exposed to S-IR and F-IR were almost p-p65 positive, but there were substantially fewer p-p65-positive cells in quercetin-pretreated mouse tongues (Figure 5(a)). Accordingly, S-IR and F-IR increased p-p65 expression in irradiated mouse tongues and the level of p-p65 expression in quercetin-pretreated mice was reduced to a level similar to that in no IR mice (Figure 5(b)). Then, we investigated the expression levels of proinflammatory cytokines. IR significantly induced proinflammatory cytokine (IL-6, IL-1*β*, TNF-*α*, TGF-*β*1, and MIP) expression in mouse tongues, and quercetin pretreatment dramatically reversed the IR-induced proinflammatory cytokine increase (Figure 5(c)). Consistent with the *in vivo* results, quercetin pretreatment reduced p-I*κ*B and p-p65 expression levels in NHKs at days 2, 5, and 7 after IR, while the total I*κ*B and p-65 levels did not change obviously in any cells (Figure 5(d)). The expression levels of proinflammatory cytokines (IL-1*β*, TNF-*α*, and TGF-*β*1) were also reduced in quercetin-pretreated NHKs at days 2, 5, and 7 after IR (Figure 5(e)). Thus, quercetin inhibits irradiation-induced activation of the NF-*κ*B pathway and the expression of downstream proinflammatory cytokines.

### 3.6. Quercetin Upregulates Bmi-1 Expression and Promotes Wound Healing

Our previous study demonstrated that BMI-1 was obviously reduced in RIOM mouse tongues at both the mRNA and protein expression levels [14]. BMI-1 plays a significant role in cellular radiosensitivity and has radioprotective effects on NHKs by silencing oxidase expression and enhancing DNA repair [18]. Therefore, we evaluated the effects of quercetin on BMI-1 expression after IR both *in vivo* and *in vitro*. BMI-1 expression was abundant in the basal layer of the oral mucosa not exposed to radiation. The number of BMI-1-positive cells was sharply decreased in S-IR and F-IR mouse oral mucosa. Quercetin-pretreated mice showed no obvious decrease in the number of BMI-1-positive cells compared with no IR mice (Figure 6(a)). Accordingly, quercetin pretreatment effectively resisted the IR-induced decrease in the protein and mRNA expression levels of BMI-1 in mouse tongues (Figures 6(b) and 6(c)). Interestingly, 2 h of quercetin treatment (5, 20, 40, 80, and 160 *μ*M) dramatically increased BMI-1 protein expression in NHKs (Figure 6(d)). BMI-1 can modulate Snail-mediated epithelial–mesenchymal transition (EMT) to promote cell migration and wound healing; therefore, we performed a wound healing assay to examine the migration ability of NHKs post-IR. Quercetin pretreatment obviously promoted NHK migration, and the healing percentages reached 43.5% and 60.2% at 24 and 48 h after IR, in contrast to 22.3% and 26.8% in control-irradiated NHKs (Figure 6(e)). Snail and Bmi-1 protein expression levels were significantly reduced at days 2, 5, and 7 after IR in irradiated NHKs but were not obviously changed in quercetin-pretreated NHKs (Figure 6(f)). These results indicate that quercetin upregulates Bmi-1 expression and promotes keratinocyte migration.

### 3.7. The Radioprotective Effects of Quercetin Are BMI-1 Dependent

To investigate whether the preventative effect of quercetin on RIOM is related to upregulating BMI-1 expression, we generated BMI-1 knockdown NHKs (NHK/shBMI-1) by infecting lentiviruses encoding BMI-1-specific shRNA sequences. The mRNA and protein expression levels of BMI-1 were significantly decreased in NHK/shBMI-1 cells, indicating that the knockdown efficiency was high (Figures 7(a) and 7(b)). We then examined whether BMI-1 silencing would repress quercetin's effect on cellular senescence induced by IR. IR induced many more senescent NHK/shBMI-1 cells than NHK/Con cells. Although quercetin pretreatment effectively reduced the number of senescent NHKs after IR, it had no effect on NHK/shBMI-1 cells (Figure 7(c)). Similarly, BMI-1 knockdown increased IR-induced p47, *γ*-H2AX, and p-p65 expression and quercetin pretreatment only inhibited the upregulation of these proteins in NHK/Con cells but not in NHK/shBMI-1 cells (Figure 7(d)). BMI-1 knockdown also increased IR-induced TGF-*β*1 and IL-1*β* mRNA expression, and quercetin pretreatment did not abolish proinflammatory factor expression after IR (Figure 7(e)). These results suggest that quercetin exerts a radioprotective effect in NHKs partially by upregulating BMI-1 expression.

## 4. Discussion

The pathogenesis of RIOM is similar in mice and humans and involves the 5 phases of initiation, primary damage, signaling amplification, ulceration, and healing. Confined to the molar protuberance, IR-induced ulceration is mainly located at the upper posterior surface of the mouse tongue and recapitulates the RIOM injury process in humans [18]. In this study, we show for the first time that quercetin pretreatment protects mice against RIOM induced by a single dose and fractionated doses of local head irradiation.

RIOM is painful and severely reduces food intake in irradiated mice, and quercetin pretreatment attenuated ulcer formation and weight loss in S-IR and F-IR mice. During RIOM development, the proliferation ability of basal epithelial cells is damaged by IR and results in tongue epithelial ablation. The basal epithelial cells are mainly keratinocytes. IR induces stress-induced premature senescence in NHKs [19]. Cellular senescence is mainly regulated by the p53/p21 and p16^INK4A^/RB signaling pathways [20, 21]. Quercetin pretreatment prevented the loss of proliferative ability of epithelial cells after IR, maintained the expression of Ki-67 and PCNA, reduced the number of senescent NHKs, and reversed the IR-induced increases in p16^INK4A^ and p21 expression. Thus, quercetin alleviates RIOM by overcoming the IR-induced cessation of proliferation.

Radiation is a form of oxidative stress to tissues and leads to ROS release from epithelial cells. Quercetin exhibits many beneficial biological properties, such as antioxidant activity. The potent antioxidant activity of quercetin due to free radical scavenging plays an important role in the prevention of oxidative damage caused by various factors [7]. Quercetin exerts antioxidant activity by regulating the activity and expression levels of antioxidant enzymes, including catalase (CAT), superoxide dismutase (SOD), glutathione S-transferase (GSH), NAD (P) H oxidase, and oxidoreductase [22–24]. IR-induced DNA damage promotes ROS generation in cells. Quercetin pretreatment reduced IR-induced cellular ROS generation and oxidative stress, as indicated by the decreased 8-OHDG expression and downregulated expression of NADPH oxidase p47. In addition, quercetin pretreatment reduced IR-induced DSBs by promoting NHEJ. Thus, quercetin pretreatment attenuates IR-induced ROS generation and DNA damage at the initiation stage of RIOM.

The NF-*κ*B pathway plays an important role in the occurrence of major damage in mucositis and provides a positive feedback loop that mediates signaling amplification [3]. ROS and DNA damage activate NF-*κ*B to stimulate the release of proinflammatory cytokines, e.g., TNF-*α*, TGF-*β*, IL-6, and IL-1*β*. Quercetin can inhibit TGF-*β* expression in irradiated mouse skin [13] and can reduce TNF-*α* expression in irradiated rat colon [12] and primary cultured dorsal root ganglion neurons [10]. Quercetin downregulates the Src/PI3K/Akt-NF-*κ*B-inflammatory pathways to attenuate atherosclerosis progression [25] and protects the skin from UVB-induced damage by inhibiting the NF-*κ*B/COX-2 signaling pathway [26]. Our results showed that quercetin pretreatment reduced TNF-*α*, TGF-*β*, IL-6, IL-1*β*, and MIP-1*β* expression in irradiated mouse tongues by inhibiting NF-*κ*B activation. Quercetin pretreatment also reduced NF-*κ*B and I*κ*B activation in irradiated NHKs, effectively alleviating TNF-*α*, TGF-*β*, and IL-1*β* expression. Thus, quercetin pretreatment reduces IR-induced NF-*κ*B activation and proinflammatory cytokine release at the primary damage and signal amplification stages of RIOM.

Keratinocyte proliferation and migration are essential for wound closure [27]. EMT is a process known to be crucial for wound healing after injury [28]. Quercetin pretreatment promoted irradiated NHK migration and maintained EMT regulator BMI-1 and Snail expression after IR, thereby accelerating reepithelialization of the oral mucosal epithelium in the healing stage of RIOM. In our previous study, we found that BMI-1 expression was decreased during RIOM pathogenesis [14]. Our data suggest that quercetin-enhanced BMI-1 expression is largely responsible for its radioprotective effects *in vitro* and *in vivo*. BMI-1, a polycomb group (PcG) protein, mediates gene silencing via chromatin remodeling and plays an important role in embryonic development [29]. BMI-1 maintains the self-renewal of stem cells and proliferation capacity by repressing p16^INK4A^, p19^Arf^, and p21 transcription [30, 31]. Although BMI-1 is abnormally highly expressed in different kinds of cancer, overexpression of BMI-1 does not lead to transformation but prolongs the life of normal cells by inhibiting cellular senescence [32, 33]. In addition, BMI-1 is a crucial factor in promoting EMT [34, 35]. Thus, upregulated BMI-1 expression by quercetin in NHKs prevents the loss of proliferation ability, reduces cellular senescence, and enhances the migration of epithelial cells after IR.

Studies have uncovered a new function of BMI-1 in DNA repair [36]. BMI-1 can maintain redox homeostasis and mitochondrial function to regulate oxidative stress levels *in vivo*, and cells derived from Bmi1(-/-) mice showed significant increases in ROS generation and DNA damage [37]. BMI-1 functions as an E3-ubiquitin ligase and promotes DNA DSB repair by ubiquitinating histone H2A and *γ*-H2AX [38, 39]. Histone ubiquitylation is critical in DSB repair through the homologous recombination (HR) and NHEJ pathways [40]. Bmi-1 reduced IR-induced ROS generation and epigenetically silenced the expression of NADPH oxidase in NHKs [18]. In the current study, the effects of quercetin pretreatment on reducing ROS generation and promoting DSB repair by the NHEJ pathway were largely related to enhanced Bmi-1 expression in NHKs.

Furthermore, our results showed that quercetin pretreatment had no radioprotective effects in BMI-1 knockdown NHKs. The senescent cell number and p47, p-p65, *γ*-H2AX, TGF-*β*, and IL-1*β* expression levels were similar in irradiated NHKs with or without quercetin pretreatment. These results demonstrate that the upregulation of BMI-1 expression by quercetin plays a key role in the preventative effects of quercetin against RIOM.

## 5. Conclusions

In this study, we provide evidence that quercetin can block multiple pathological processes of RIOM and exert preventive effects in irradiated mice. Quercetin also exerted radioprotective effects in NHKs partially by upregulating BMI-1 expression (Figure 8). Hence, quercetin is a potential treatment option for preventing RIOM and should be further explored for its therapeutic effect on RIOM.

## Figures and Tables

**Figure 1:** Quercetin attenuates radiation-induced ulcer formation. (a) Mouse body weight changes in the S-IR, S − IR + QCT, F-IR, and F − IR + QCT groups after IR (*n* = 5). ^∗^*P* < 0.05, ^∗∗^*P* < 0.01, and ^∗∗∗^*P* < 0.001 vs. IR mice. (b) Mouse tongues were obtained at day 9 after IR and were stained with TB to observe the formation of ulcers. The ulcers are marked by yellow circles. (c) Quantification of the tongue ulcer diameter shown in (b), ^∗∗∗^*P* < 0.001 vs. IR mice (*n* = 5). (d) HE staining of mouse tongues shows the structure of the oral mucosa obtained at day 9 after IR. Scale bars, 100 *μ*m.

**Figure 2:** Quercetin maintains proliferative activity and reduces cellular senescence after IR. (a) IHC staining of Ki-67 in tongue tissues harvested at day 9 after IR. Scale bars, 100 *μ*m. (b) Western blot analysis of PCNA expression in mouse tongues (*n* = 3). (c) Western blot analysis of p21 expression in mouse tongues (*n* = 3). (d) The relative mRNA expression levels of p16^INK4A^ and p21 in mouse tongues were detected by qPCR. ^∗∗^*P* < 0.01 and ^∗∗∗^*P* < 0.001 vs. nonirradiated control mice. (e) Cellular senescence was measured in NHKs at days 0, 2, 5, and 7 after IR by SA-*β*-Gal assay. (f) The numbers of SA-*β*-Gal-positive NHKs were counted. ^∗∗∗^*P* < 0.001 vs. control NHKs. Scale bar, 50 *μ*m. (g) Quercetin-pretreated NHKs showed less radiosensitivity than control NHKs by colony formation assay. (h) Western blot analysis of PCNA and p21 expression in NHKs at days 0, 2, 5, and 7 after IR.

**Figure 3:** Quercetin attenuates IR-induced ROS generation. (a) Mouse tongues were obtained at day 9 after IR, and frozen sections were stained with DHE to observe the formation of ROS. Scale bars, 200 *μ*m. (b) IHC staining of 8-OHDG of tongue tissues. Scale bars, 100 *μ*m. (c) Western blot analysis of p47 expression in mouse tongues (*n* = 3). (d, e) NHKs with/without quercetin pretreatment were stained with DHE at day 7 after IR, and the fluorescence intensity of DHE was quantified by flow cytometry. ^∗∗∗^*P* < 0.001. (f) Western blot analysis of p47 expression in control and quercetin-pretreated NHKs at days 0, 2, 5, and 7 after IR.

**Figure 4:** Quercetin mitigates DNA damage induced by IR. (a) IHC staining of *γ*-H2AX in tongue tissues harvested at day 9 after IR. Scale bars, 100 *μ*m. (b) Western blot analysis of *γ*-H2AX expression in mouse tongues (*n* = 3). (c) Control and quercetin-pretreated NHKs were stained with the *γ*-H2AX antibody (red) at 6 h after IR, and the number of *γ*-H2AX foci per cell was counted and statistically analyzed. ^∗∗∗^*P* < 0.001. (d) Western blot analysis of *γ*-H2AX expression in NHKs at days 0, 2, 5, and 7 after IR. (e) A neutral comet assay was performed in NHKs at 6 h after IR, and DNA DSBs were quantitated by the length of the DNA tail. ^∗∗∗^*P* < 0.001. (f) Deletion distributions in NHEJ of AAVS1 cuts between NHKs. The median deletion length analysis shows a shift toward shorter deletions in quercetin-pretreated NHKs. ^∗∗∗^*P* < 0.001 vs. control NHKs. (g) Frequency of deletions with different deletion lengths among NHEJs in NHKs.

**Figure 5:** Quercetin inhibits IR-induced NF-*κ*B activation and proinflammatory cytokine production. (a) IHC staining of p-p65 (Ser536) in tongue tissues harvested at day 9 after IR. Scale bars, 100 *μ*m. (b) Western blot analysis of p-p65 (Ser536) expression in mouse tongues (*n* = 3). (c) The relative mRNA expression levels of IL-6, IL-1*β*, TNF-*α*, TGF-*β*1, and MIP-1*β* were measured by qPCR in mouse tongues (*n* = 5). ^∗∗^*P* < 0.01 and ^∗∗∗^*P* < 0.001. (d) Western blot analysis of p-p65 (Ser536), NF-*κ*B, p-I*κ*B (Ser32/36), and I*κ*B expression in NHKs at 0, 2, 5, and 7 days after IR. (e) The relative mRNA expression levels of IL-1*β*, TGF-*β*1, and TNF-*α* in NHKs at 0, 2, 5, and 7 days after IR were measured by qPCR. ^∗^*P* < 0.05, ^∗∗^*P* < 0.01, and ^∗∗∗^*P* < 0.001 vs. control NHKs.

**Figure 6:** The radioprotective effects of quercetin are related to upregulating BMI-1 expression. (a) IHC staining of BMI-1 in tongue tissues harvested at day 9 after IR. Scale bars, 100 *μ*m. (b) Western blot analysis of BMI-1 expression in mouse tongues (*n* = 3). (c) The relative mRNA expression levels of BMI-1 were measured by qPCR in mouse tongues (*n* = 5). ^∗∗∗^*P* < 0.001. (d) Western blot analysis of BMI-1 expression in NHKs pretreated with the indicated doses of quercetin for 2 h. (e) A wound healing assay was performed in control and quercetin-pretreated NHKs after 5 Gy IR. Images were taken at 0, 24, and 48 h after irradiation, and then, the healing percentages of NHKs were quantified. ^∗∗∗^*P* < 0.001 vs. control NHKs. (f) Western blot analysis of BMI-1 and Snail expression levels in NHKs at 0, 2, 5, and 7 days after IR.

**Figure 7:** The radioprotective effects of quercetin are BMI-1 dependent. (a) *BMI-1* was knocked down using lentiviral shRNA in NHKs. *BMI-1* expression levels were decreased in NHK/sh-BMI-1 cells. ^∗∗∗^*P* < 0.001. (b) BMI-1 expression levels were decreased in NHK/sh-BMI-1 cells. (c) Cellular senescence was measured in NHKs at day 5 after IR by SA-*β*-Gal assay. The numbers of SA-*β*-Gal-positive NHKs were counted. ^∗∗^*P* < 0.01 and ^∗∗∗^*P* < 0.001. Scale bar, 50 *μ*m. (d) Western blot analysis of p47, *γ*-H2AX, p65, p-p65 (Ser536), and BMI-1 expression in NHKs at day 5 postirradiation. (e) The relative mRNA expression levels of TGF-*β*1 and IL-1*β* were measured by qPCR in NHKs at day 5 postirradiation. ^∗^*P* < 0.05, ^∗∗^*P* < 0.01, and ^∗∗∗^*P* < 0.001.

**Figure 8:** Schematic representation of the possible molecular mechanism by which quercetin prevents RIOM. The pathogenesis of RIOM includes the initiation, primary damage, signaling amplification, ulceration, and healing phases. Quercetin alleviates ROS generation, NF-*κ*B pathway activation, and downstream proinflammatory cytokine production and reduces DNA double-strand breaks (DSBs) and cellular senescence induced by IR. Quercetin maintains the cell proliferation ability and promotes EMT. Thus, quercetin attenuates multiple pathological processes of RIOM partially by upregulating BMI-1 expression.

## Data Availability

All data generated or analyzed during this study are included in this published article. Supplementary data for this article can be found in the online version.

## Supplementary Materials

Supplementary materials Figure S1: Effect of quercetin on the proliferation of NHKs. The survival of NHKs was detected by CCK8 assay after treatment with different doses of quercetin (0–20 *μ*M) for 24 h. ^∗^*P* < 0.05 and ^∗∗∗^*P* < 0.001 vs. control cells. Table S1: Primary antibodies for Western blot, IF, and IHC. Table S2: Primer sequences for quantitative RT-PCR. Table S3: Clonogenic survival parameters fitting the data to a multitarget model.
